# Prevalence and Antimicrobial Susceptibility of *Streptococcus pneumoniae* Isolated from Clinical Samples in the Past 8 Years in Korea

**DOI:** 10.1155/2021/6615334

**Published:** 2021-04-28

**Authors:** Jae Soo Kim, Bo Kyeung Jung, Jong Wan Kim, Ga Yeon Kim

**Affiliations:** ^1^Department of Laboratory Medicine, Dankook University Hospital, 119 Dandae-ro, Dongnan-Gu, Cheonan-Si, Chungnam 31116, Republic of Korea; ^2^Department of Laboratory Medicine, Dankook University College of Medicine, 119 Dandae-ro, Dongnan-Gu, Cheonan-Si, Chungnam 31116, Republic of Korea; ^3^Department of Public Health, Dankook University Graduate School, 119 Dandae-ro, Dongnan-Gu, Cheonan-Si, Chungnam 31116, Republic of Korea

## Abstract

Pneumococcal infection is the main causative agent of pneumonia, meningitis, and sepsis in immunocompromised and elderly people. The samples in this study were collected from subjects in an 800-bed hospital in Chungnam province, Korea, over the past 8 years. Of the 473,230 samples obtained for microbial culture from 2012 to 2019, *Streptococcus pneumoniae* was isolated from 714 samples collected from 702 patients, with a pneumococcal-positive rate of 0.15%. We investigated the temporal, demographic, and specimen-specific distributions, as well as the antibiotic susceptibility pattern for *S. pneumonia*. The age of patients ranged from 0 days to 98 years, with an average age of 64.7 years. The distribution among the sexes was 2.4 : 1 (male : female), with more samples isolated from male patients. We observed that spring was the predominant season in which the infection occurred, accounting for 37.6% of the cases. Pneumococci were most frequently isolated from sputum (608 cases, 85.2%). Invasive infections were detected at a rate of 66% (in blood cultures), and noninvasive infections were detected at a rate of 91% (in sputum cultures). Antimicrobial resistance to ceftriaxone, cefotaxime, erythromycin, tetracycline, clindamycin, cotrimoxazole, levofloxacin, and penicillin, based on noninvasive infections, was observed in 21.6%, 27.2%, 79.2%, 73.2%, 68.0%, 51.3%, 9.8%, and 18.1% of cases, respectively. Additionally, on average, 66.9% of multidrug-resistant bacteria showed resistance to three or more antimicrobial agents, and 2.8% showed resistance to all other antibacterial agents except vancomycin. These results might facilitate the administration of appropriate empirical antibacterial therapy for pneumococcal infections.

## 1. Introduction

*Streptococcus pneumoniae* is a gram-positive facultative anaerobic bacterium, which exhibits partial hemolysis under aerobic conditions or complete hemolysis under anaerobic conditions [1]. These bacteria are generally diplococcal and do not undergo sporulation or exhibit motility (“*Streptococcus pneumoniae*,” http://microbewiki.kenyon.edu. Retrieved October 24, 2017). They are also sensitive to optochin, and thus, an optochin test can be performed to distinguish them from *Viridans streptococci*, another strain that exhibits *α*-hemolysis; however, optochin resistance has recently been reported in *S. pneumoniae* [2]. *S. pneumoniae* can also be differentiated through bile solubility testing based on its sensitivity to bile dissolution. These capsule-forming gram-positive bacteria display a unique diplococcal conformation in a lancet shape upon gram staining. They also possess polysaccharide capsules that act as a toxin towards organic bodies. According to the antigenicity of their capsular polysaccharides, almost 100 serotypes have been identified. These serotypes show varying levels of toxicity, prevalence rates, and drug resistance patterns. The main toxic factors are pneumolysin, antiphagocytic capsule, various adhesins, and immunogenic cell wall components [3–5]. When the air sacs in the lungs are inhabited by *S. pneumoniae*, an inflammatory response is activated in the body to promote the influx of plasma, serum, and leukocytes, which subsequently fill the alveoli, a state referred to as pneumonia [6].

*S. pneumoniae* is generally found in the respiratory, paranasal, and nasal cavities, where they cause no symptoms in healthy individuals. However, in children and the elderly with a reduced level of immunity, these species are the main causal agents of pneumonia, meningitis, and sepsis, in addition to causing diseases other than pneumonia [7]. An invasive pneumococcal infection is diagnosed when *S. pneumoniae* is isolated from physiologically bacteria-free areas, such as the blood and cerebrospinal fluid. The presence of *S. pneumoniae* in these areas causes diseases, such as sepsis, cerebromeningitis, osteomyelitis, septic arthritis, endocarditis, pericarditis, peritonitis, and brain abscess [8]. However, in noninvasive infections, including sinusitis, acute tympanitis, and local community-acquired pneumonia, which account for most pneumococcal infections, the *S. pneumoniae* test is not typically performed; thus, such difficulties in defining the cause of *S. pneumoniae*-related conditions prevent the calculation of their incidence rates. According to previous studies, *S. pneumoniae* is thought to cause 15–43% of local community-acquired pneumonia cases and 30–35% of acute tympanitis cases [9].

In 2003, the 7-valent pneumococcal protein conjugate vaccine (PCV7) was introduced to Korea as an optional vaccine for children under 5 years of age. In March 2010, PCV10 (against serotypes 4, 6B, 9V, 14, 18C, 19F, 23F, 1, 5, and 7F) and PCV13 (against serotypes 4, 6B, 9V, 14, 18C, 19F, 23F, 1,5, 7F, 3, 6A, and 19A) were introduced in Korea^1^, and in 2014, the pneumococcal vaccine was included in the national vaccination program (4^th^ vaccination for 2 months, 4 months, 6 months, and 12-15 months after birth).

The statistics for the year 2012 for the causes of mortality in Korea show that mortality due to pneumonia was 20.5 per 100,000 individuals, with the disease ranking sixth among all causes of mortality and first for infectious diseases [10]. The causes of pneumonia vary with different bacteria and viruses, and although the early detection of causal bacteria is a prerequisite for selecting suitable antibiotics, they are identified in only 35–60% of cases; thus, patients are administered empirical antibiotic treatment [11]. Therefore, analysing the distribution and pattern of antibiotic resistance of *S. pneumoniae* will provide an improved basis for its treatment.

Therefore, investigating patterns of changes in the antimicrobial susceptibility of *S. pneumoniae* is essential to select a suitable antimicrobial agent or to monitor and control emerging new resistant bacterial species in clinical practice. The pattern of antimicrobial resistance might differ by varying degrees according to the region and time. This study was conducted to determine the trends in the isolation frequency and antimicrobial susceptibility of *S. pneumoniae* based on yearly/seasonal prevalence, age, sex, specimen-specific distributions, and invasiveness factors. *S. pneumoniae* was isolated from patients at an 800-bed university hospital in the Chungcheong province between 2012 and 2019. These findings can be used to identify suitable empirical antimicrobial therapies to treat pneumococcal infections.

## 2. Materials and Methods

### 2.1. Subjects

The study included 714 cultured *S. pneumoniae* strains that had been isolated from 473,230 patients at an 800-bed university hospital located in Chungnam over the past 8 years, for which a request had been made to the Department of Laboratory Medicine. The study included the period between January 2012 and December 2019. At the time of the study, the 702 confirmed patients were divided by age into infants (<1 year), children (1–18 years), and adults (>18 years), with a median age of 64.7 years (0–98 years). The Institutional Review Board Deliberations of Dankook University approved this study (IRB No. DKU 202001014). The need for informed consent was waived as this study does not use personally identifiable information of any subject.

### 2.2. Testing Methods

The samples for which a culture request had been made were inoculated onto blood agar plates, which were then cultured at 36°C and 5% CO_2_ in an incubator for 18–24 h. Among the cultured colonies, *S. pneumoniae* formed colonies that were 1–1.5 mm in diameter with a flat, dent-centred, green hemolytic band on the blood agar plate. In sputum samples, to distinguish streptococcal species from the normal flora, an optochin test was performed, and strains exhibiting a zone of inhibition ≥ 14 mm were used in the test. The Bact/Alert 3D (bioMérieux, Marcy-l'Étoile, France) incubator was used for blood cultures. SA medium (aerobic), which is a trypticase soy broth, and SN medium (anaerobic), which is a thioglycolate broth for adults, were also used. PF medium was used for *S. pneumoniae* isolated from children and infants. The cultures were incubated for up to 5 days. Samples from pus, throat, and reproductive organs were collected using sterilised swabs and immersed in Stuart transport medium for storage at 4°C until analysis. All samples, except that from blood, were inoculated onto blood agar and MacConkey agar plates as soon as possible and then cultured at 36°C and 5% CO_2_ in an incubator. Urine samples were inoculated using a 1 *μ*L standard platinum loop.

Each bacterial colony grown on the medium was identified using the VITEK2 (bioMérieux) GP card and adjusted to a McFarland standard of 0.5 in 0.45% phosphate-buffered saline. For the antimicrobial susceptibility tests, the ST03 card was used with the following nine antibiotics: penicillin, erythromycin, cefotaxime, ceftriaxone, clindamycin, tetracycline, cotrimoxazole, levofloxacin, and vancomycin. To measure the minimal inhibitory concentration (MIC), the broth microdilution method was performed as described in the Clinical and Laboratory Standards Institute (CLSI) M100-S29 [7]. Additionally, to determine antibiotic resistance rates, susceptibility-free cases of moderate resistance and high resistance were included.

In cases of central nervous system (CNS) infection with *S. pneumoniae*, penicillin susceptibility (≤0.06 *μ*g/mL), intermediate susceptibility (0.12–1.0 *μ*g/mL), and resistance (≥2 *μ*g/mL) were determined. In cases of non-CNS infection, the CLSI standards for penicillin susceptibility (≤2 *μ*g/mL), intermediate susceptibility (4 *μ*g/mL), and resistance (≥8 *μ*g/mL) were applied. If resistance to three or more antibiotics was observed (penicillin, lincosamide, macrolide, cephalosporin, fluoroquinolone, glycopeptide, cotrimoxazole, and tetracycline), the case was defined as multidrug-resistant, among which cases of intermediate resistance were not included. Statistical analysis was performed using MS Excel (Microsoft, Redmond, WA, USA) and SPSS Statistical Procedure for Windows (SPSS PASW Statistic 23.0, SPSS Inc., Chicago, IL, USA). Using frequency analysis and graphs, distribution patterns of *S. pneumoniae* isolated from clinical specimens were confirmed by year and month of infection and age of patients, and seasonal differences were statistically verified by *t*-testing (*P* < 0.05).

For cases in which *S. pneumoniae* was isolated multiple times from a single patient, the first test was included in the analysis. For cases in which *S. pneumoniae* simultaneously presented invasive and noninvasive infections in culture, the two cases were separately analysed. Invasive infections included cases of *S. pneumoniae* isolation from blood, cerebrospinal fluid, pleural fluid, peritoneal fluid, and bile, whereas noninvasive infections included cases isolated from sputum, ear, eye, pus, and urine. For distributions associated with yearly and monthly (seasonal), age/sex of patient, and specimen, invasive and noninvasive pneumonia was separately tested via antimicrobial susceptibility tests, and the MIC method was used to investigate the trends in antimicrobial susceptibility.

## 3. Results

### 3.1. Yearly Distribution

Among the 473,230 samples for which microbial cultures were requested during the period between 2012 and 2019, we isolated *S. pneumoniae* from 714 samples obtained from 702 patients, which had a pneumococcal-positive rate of 0.15%. The yearly isolation frequency of *S. pneumoniae* showed a gradual decrease from 104 in 2012 to 77 in 2018 and a rapid increase to 113 in 2019. The lowest isolation frequency was 70 in 2014 (Figure 1).

### 3.2. Monthly or Seasonal Distribution

For the monthly distribution, the highest number of cases was 93 (13.2%) in March, followed by 87 (12.4%) in April and 83 (11.8%) in May. In contrast, the lowest number of cases was 23 (3.3%) in September, followed by 30 (4.3%) in October and 39 (5.6%) in August. For the seasonal distribution, the highest number of cases was 263 (37.5%) in spring, followed by 207 (29.5%) in winter and 131 (18.7%) in summer, whereas the lowest number of cases was 101 (14.4%) in autumn (Figure 2). Spring was ranked as the season with the highest isolation rates compared with other seasons (*P* < 0.05); however, the difference in rates between summer and autumn was not statistically significant (*P* = 0.148).

### 3.3. Distribution by Age and Sex

At the time of the study, the age distribution ranged from 0 days to 98 years, with the average age of patients being 64.7 years. The number of cases was nine (1.3%) in infants < 1 year, 19 (2.7%) in children aged 1–18 years, and 674 (96.0%) in adults ≥ 18 years. Among the adults, the elderly (≥60 years) accounted for most cases (71.6%), and the sex distribution was 2.4 : 1 (male : female), indicating a higher number of cases in male patients (Table 1).

### 3.4. Distribution by Specimen Type

*S. pneumoniae* was most frequently isolated from the sputum (608 cases; 85.2%), followed by blood (33 cases; 4.6%), ear (16 cases; 2.2%), cerebrospinal fluid (seven cases; 1.0%), and other areas (50 cases; 7.0%). The total number of cases was 714 (Figure 3).

### 3.5. Distribution according to Invasiveness

For invasive infections, the highest isolation frequency was 66% from the blood, followed by cerebrospinal fluid, pleural fluid, and peritoneal fluid. For noninvasive infections, the highest isolation frequency was 91% from the sputum, followed by ear, eye, wounds, and urine. The overall specimen-specific distributions of the isolates were as follows: sputum in 598 cases (85%), blood in 31 cases (4.4%), ear in 16 cases (2.3%), cerebrospinal fluid in seven cases (1.0%), and urine in six cases (0.9%) (Table 2). The clinical symptoms in patients harboring the *S. pneumoniae* isolates obtained from invasive specimens (*n* = 49) are shown in Table 3.

### 3.6. Antimicrobial Susceptibility Testing Results

Antimicrobial susceptibility by year was analysed separately for invasive and noninvasive infections. For invasive infections, the cases of CNS infection and non-CNS infection were separately analysed. In cases of invasive infections, CNS infection-causing *S. pneumoniae* isolates showed a high penicillin resistance rate of 85.7% (Table 4), whereas non-CNS infection-causing *S. pneumoniae* isolates were associated with a relatively low resistance rate of 13.9% (Table 5). The resistance rate was 18.9% for noninvasive infection-causing *S. pneumoniae* isolates (Table 6). This might be because penicillin susceptibility was divided according to resistance rates of ≤0.06 *μ*g/mL, 0.12–1.0 *μ*g/mL, and ≥2 *μ*g/mL for *S. pneumoniae* CNS infections, whereas the standards of the CLSI Guidelines for penicillin susceptibility were ≤2 *μ*g/mL, 4 *μ*g/mL, and ≥8 *μ*g/mL for non-CNS infections. In the case of noninvasive infections, the resistance rates were relatively low, specifically 16.7% in 2012, 11.6% in 2014, 15.6% in 2015, 15.7% in 2017, and 16.2% in 2019; however, relatively high rates were also observed, such as 20% in 2013, 19.9% in 2016, and 26% in 2018 (Figure 4).

Resistance to three or more of the following antibiotics was observed: penicillin, macrolide, clindamycin, cephalosporin, fluoroquinolone, chloramphenicol, tetracycline, and cotrimoxazole; these were defined as multidrug-resistant cases (MDR). During the study period, MDR was detected in 472/706 cases (66.9%), with the highest value of 62/86 cases (72.1%) in 2013 and the lowest value of 42/82 cases (51.2%) in 2017. Among these, MDR including resistance to all antimicrobial agents except vancomycin occurred in 20/706 (2.8%) cases during the study period (Figure 5).

Antimicrobial susceptibility testing was carried out for 10 antibiotics, including penicillin, erythromycin, cefotaxime, ceftriaxone, clindamycin, tetracycline, cotrimoxazole, levofloxacin, vancomycin, and linezolid; however, no samples showed resistance to vancomycin or linezolid, and the test included results only for vancomycin. All of these samples were isolated from the sputum. Four antibiotics, namely, cefotaxime, clindamycin, erythromycin, and tetracycline, were associated with the lowest resistance rate in 2017, as was observed in cases of MDR, which showed a steady decrease from 72.1% in 2013 to 51.2% in 2017, followed by a steep increase to 68.4% in 2018 and the lowest value of 70% in 2019. According to the analysis of invasiveness, resistance to erythromycin, cefotaxime, and ceftriaxone in nonmeningeal invasive infections was observed in 69.4%, 19.5%, and 16.6% of cases, respectively (Table 5). For noninvasive infections, the resistance rates were even higher at 80.2%, 27.8%, and 22.0%, respectively (Table 6), whereas resistance to other antimicrobial agents was also high primarily in noninvasive infections.

## 4. Discussion

*S. pneumoniae* shows resistance to *β*-lactam antibiotics based on a mechanism whereby a penicillin-binding protein undergoes structural changes that reduce its affinity to penicillin, whereas the resistance to macrolide antibiotics is known to be based on the inhibition of ribosome binding to prevent drug penetration and accumulation [12–14]. In Korea, the first case of penicillin-resistant *S. pneumoniae* was reported in the early 1980s; the reported rate of resistance was approximately 40–60% in the early 1990s and approximately 60–80% in the late 1990s [15]. We observed the highest resistance rate of 79.2% to erythromycin, a macrolide antibiotic, which was determined to be the result of the frequent use of this drug in empirical treatments.

The penicillin susceptibility criteria of CLSI for *S. pneumoniae* were updated from an MIC of 0.06 to 2 *μ*g/mL for nonmeningeal infections in 2018 [16, 17]. In contrast to studies applying the criteria set before 2008, studies of nonmeningeal, invasive pneumococcal infections based on the revised penicillin susceptibility criteria set after 2008 predicted increased penicillin susceptibility. In fact, among the 123 invasive pneumococcal species identified across eight university hospitals in Korea between 2006 and 2010, 91.1% of isolates showed a penicillin MIC ≤ 2 *μ*g/mL, indicating penicillin susceptibility [18]. Thus, prior to the extensive use of antibiotics as an empirical treatment for nonmeningeal invasive pneumococcal infection in children and adolescents in Korea, the use of *β*-lactam antibiotics, including penicillin, as an early empirical antibiotic might be recommended [19, 20].

The resistance rates of *S. pneumoniae* isolated at primary and secondary medical institutions in Korea from July 2009 to December 2013, as reported by the KCDC, were 28.7%, 25.9%, 84.3%, 78.7%, 68.5%, 57.4%, 1.9%, and 35.2% (high resistance rate 8.3% and intermediate rate 26.9%) to ceftriaxone, cefotaxime, erythromycin, tetracycline, clindamycin, cotrimoxazole, levofloxacin, and penicillin, respectively, with 79.6% MDR bacteria [21]; however, in this study, for noninvasive infections, the resistance rates were 21.6%, 27.2%, 79.2%, 73.2%, 68.0%, 51.3%, 9.8%, and 18.1% (high resistance rate 7.1% and intermediate rate 11.0%), respectively, with 65.0% MDR bacteria, indicating a high level of resistance. Nonetheless, the resistance rate was lower than that in the 2014 KCDC reports from primary and secondary medical institutions, with the penicillin resistance rate showing a particularly notable difference. The levofloxacin resistance rate, however, was 9.8%, which was higher than that previously reported at primary and secondary medical institutions. This might be because of the generally larger number of prescriptions of antimicrobial agents at primary and secondary medical institutions. In this study targeting a tertiary medical institution, the administration of levofloxacin as a quinolone-based antibiotic with a low level of resistance was relatively more frequent. In addition, the antimicrobial resistance of *S. pneumoniae* isolated from patients with regional pneumonia at primary and secondary medical institutions was considerably higher than that in the institution targeted in this study with respect to the rate of single-drug resistance and MDR. This could be because the patients had been administered empirical antibiotic treatment beforehand, rather than treatments focused on the causal bacteria, as it is often difficult to identify the precise cause of regional pneumonia for which the causal bacteria might vary. Thus, for pneumococcal infections, the choice of antibiotics is extremely limited, necessitating an examination of the current state of antibiotic resistance rates of *S. pneumoniae* in Korea through continuous monitoring.

According to previous reports, pneumococcal infections most commonly occur during the season with the highest incidence of respiratory infections. Similarly, we observed the highest number of cases (263 cases; 37.5%) in spring, followed by 207 cases (29.5%) in winter and 131 cases (18.7%) in summer, with the lowest number of cases (101 cases; 14.4%) in autumn. The average proportion of MDR bacteria, showing resistance to three or more antimicrobial agents, was 65.0% in this study, with the highest resistance rate of 72.1% in 2013 and the lowest rate of 51.2% in 2017. Among them, 20 cases (2.8%) showed resistance to all antimicrobial agents excluding vancomycin.

A limitation of this study was that we were unable to identify the serotypes of the specimens using multiplex PCR, particularly the 49 invasive specimens. However, a review of the available literature [22] revealed the existence of an effect of the pneumococcal vaccine on the distribution of serotypes, which may be applicable to the Cheonan province of Korea. Invasive pneumococcal disease (IPD) is not classified as a nationally notifiable disease in Korea, and population-based data on the incidence of this disease are not available, making it difficult to determine the efficacy of the vaccine. However, since the introduction of PCV, there have been reports on the altered incidence of pneumococcal disease. Forty-nine cases (which includes 44 patients) of invasive infections in this study involved patients of ages in the range 43 to 86 years, excluding one 20-month-old female and a 23-year-old male (24 subjects were over 65 years old). All the 49 cases in this study involved adults 18 years of age or older, except for one case. There is no confirmed data on whether the 49 subjects were vaccinated, although vaccination was mandatory for infants since 2014. According to a study [23], after PCV10 and PCV13 were introduced in Korea in 2010, PCV7 serotypes constituted 9.3% of IPD and PCV13 serotypes constituted 53.3% of all IPD from 2011 to 2013, whereas serotypes 1, 5, and 7F were absent. Serotype 19A accounted for 32% of the total IPD, whereas serotype 6A accounted for 5.3%. Other common *S. pneumoniae* serotypes were 10A, 15A, 15B, 15C, 23A, and 11A. According to this result, during the period of this study (2012 to 2019), it can be expected that the rate of PCV13 serotypes such as 19A would have decreased as the rate of administration of PCV13 vaccine increased. Additionally, nonvaccine serotypes may relatively increase in unvaccinated patients due to herd effect or herd immunity. According to another study [24], statistically significant highly invasive *S. pneumoniae* serotypes include the following 20 types: 1, 3, 4, 5, 6B, 7F, 8, 9N, 9L, 9V, 9A, 12B, 12F, 14, 18, 18C, 19A, 20, 22F, and 33F.

## 5. Conclusions

In this study, we examined the temporal, demographic, and specimen-specific distribution, as well as antibiotic susceptibility pattern, for *S. pneumoniae* isolated from patients at a tertiary medical institution in Chungnam over the past 8 years. Based on our findings, suitable empirical antimicrobial therapies against pneumococcal infections could be determined.

## Figures and Tables

**Figure 1:** Yearly distribution of *Streptococcus pneumoniae* by age.

**Figure 2:** Monthly and seasonal distribution of 714 pneumococcal infections over eight consecutive years. Spring season is defined as the period including the months of March, April, and May, and summer is defined as the period including the months of June, July, and August. Autumn is defined as the period including the months of September, October, and November, and winter includes December, January, and February. *P* < 0.05 is considered statistically significant.

**Figure 3:** Distribution of specimen types associated with *Streptococcus pneumoniae* infection over a period of eight consecutive years.

**Figure 4:** Antimicrobial resistance (%) of *Streptococcus pneumoniae* isolates obtained in each year. MDR: multidrug resistance.

**Figure 5:** Multidrug resistance (MDR) segregation frequency by year. The number after MDR is the number of antibiotics to which resistance was observed. N MDR: resistant to fewer than three antibiotics.

**Table 1:** Age and sex distribution of the subjects of the study.

Age group	Male (%)	Female (%)	Total (%)
<1	6 (0.85)	3 (0.43)	9 (1.3)
1–18	10 (1.4)	9 (1.3)	19 (2.7)
>18	482 (68.7)	192 (27.4)	674 (96.0)
Total (%)	498 (70.9)	204 (29.1)	702 (100)

**Table 2:** Distribution of *Streptococcus pneumoniae* isolates by clinical specimens for disease invasiveness.

	Specimen	No. of isolates (%)
Invasive (*n* = 49)	Blood	33 (4.6)
	CSF	7 (1.0)
	PF	4 (0.6)
	AF	3 (0.4)
	JF	1 (0.1)
	Bile	1 (0.1)
Noninvasive (*n* = 665)	Sputum	608 (85.2)
	Ear	16 (2.2)
	Eye	3 (0.4)
	Pus	5 (0.7)
	Urine	6 (0.8)
	Other	27 (3.8)
	Total	714 (100)

**Table 3:** The clinical symptoms from all isolates of *S. pneumonia* obtained from invasive specimens.

Clinical symptoms	No. of isolates (%)
Pneumonia	24 (48.9)
Meningitis	10 (20.4)
Cancer	6 (12.2)
Bacterial peritonitis	3 (6.1)
Liver cirrhosis with ascites	3 (6.1)
Etc.	3 (6.1)
Total	49 (100)

**Table 4:** Antimicrobial susceptibility (%) pattern of *Streptococcus pneumoniae* isolated from meningitis patients among invasive specimens.

Antimicrobial agents	No. of isolates	Resistant		Intermediate		Susceptible	
		% of isolates	MIC breakpoints (*μ*g/mL)	% of isolates	MIC breakpoints (*μ*g/mL)	% of isolates	MIC breakpoints (*μ*g/mL)
Clindamycin	7	57.1	≥1	0	0.5	42.9	≤0.25
Cefotaxime	7	18.6	≥2	27.9	1	53.5	≤0.5
Ceftriaxone	7	28.6	≥2	57.1	1	14.3	≤0.5
Erythromycin	7	57.1	≥1	0	0.5	42.9	≤0.25
Levofloxacin	7	0	≥8	0	4	100	≤2
Penicillin G	7	85.7	≥0.12	0	—	14.3	≤0.06
Cotrimoxazole	7	28.6	≥4/76	0	1/19~2/38	71.4	≤0.5/9.5
Tetracycline	7	57.1	≥4	0	2	42.9	≤1
Vancomycin	7	0	—	0	—	100.0	≤1

**Table 5:** Antimicrobial susceptibility (%) pattern of *Streptococcus pneumoniae* isolated from nonmeningitis patients among invasive specimens.

Antimicrobial agents	No. of isolates	Resistant		Intermediate		Susceptible	
		% of isolates	MIC breakpoints (*μ*g/mL)	% of isolates	MIC breakpoints (*μ*g/mL)	% of isolates	MIC breakpoints (*μ*g/mL)
Clindamycin	36	66.7	≥1	0	0.5	33.3	≤0.25
Cefotaxime	36	2.8	≥4	16.7	2	80.5	≤1
Ceftriaxone	36	8.3	≥4	8.3	2	83.3	≤1
Erythromycin	36	69.4	≥1	0	0.5	30.6	≤0.25
Levofloxacin	36	5.6	≥8	2.8	4	91.7	≤2
Penicillin G	36	2.8	≥8	11.1	4	86.1	≤2
Cotrimoxazole	36	30.6	≥4/76	8.3	1/19~2/38	61.1	≤0.5/9.5
Tetracycline	36	75.0	≥4	0	2	25.0	≤1
Vancomycin	36	0	—	0	—	100.0	≤1

**Table 6:** Antimicrobial susceptibility (%) pattern of *Streptococcus pneumoniae* isolated from noninvasive specimens.

Antimicrobial agents	No. of isolates	Resistant		Intermediate		Susceptible	
		% of isolates	MIC breakpoints (*μ*g/mL)	% of isolates	MIC breakpoints (*μ*g/mL)	% of isolates	MIC breakpoints (*μ*g/mL)
Clindamycin	644	67.2	≥1	0.9	0.5	31.9	≤0.25
Cefotaxime	651	13.7	≥4	14.1	2	72.2	≤1
Ceftriaxone	650	14.8	≥4	7.2	2	78.0	≤1
Erythromycin	636	79.7	≥1	0.5	0.5	19.8	≤0.25
Levofloxacin	651	9.1	≥8	0.9	4	90.0	≤2
Penicillin G	655	7.9	≥8	11.0	4	81.1	≤2
Cotrimoxazole	655	40.8	≥4/76	11.4	1/19~2/38	47.8	≤0.5/9.5
Tetracycline	650	72.3	≥4	0.9	2	26.8	≤1
Vancomycin	655	0	—	0	—	100.0	≤1

## Data Availability

The statistical data used to support the findings of this study are available from the corresponding author upon request. The relevant raw data will be made available to researchers wishing to use them for noncommercial purposes.

## References

[1] Ryan K. J., Ray C. G. (2004). *Sherris Medical Microbiology*.

[2] Pikis A., Campos J. M., Rodriguez W. J., Keith J. M. (2001). Optochin resistance in Streptococcus pneumoniae: mechanism, significance, and clinical implications. *Journal of Infectious Diseases*.

[3] Hausdorff W. P., Feikin D. R., Klugman K. P. (2005). Epidemiological differences among pneumococcal serotypes. *The Lancet Infectious Diseases*.

[4] Hausdorff W. P., Bryant J., Paradiso P. R., Siber G. R. (2000). Which pneumococcal serogroups cause the most invasive disease? Implications for conjugate vaccine formulation and use: part I. *Clinical Infectious Diseases*.

[5] Hausdorff W. P., Bryant J., Kloek C., Paradiso P. R., Siber G. R. (2000). The contribution of specific pneumococcal serogroups to different disease manifestations: implications for conjugate vaccine formulation and use, part II. *Clinical Infectious Diseases*.

[6] Niu C., Yu D., Wang Y. (2013). Common and pathogen-specific virulence factors are different in function and structure. *Virulence*.

[7] Van de Beek D., de Gans J., Tunkel A. R., Wijdicks E. F. M. (2006). Community-acquired bacterial meningitis in adults. *New England Journal of Medicine*.

[8] Siemieniuk R. A. C., Gregson D. B., Gill M. J. (2011). The persisting burden of invasive pneumococcal disease in HIV patients: an observational cohort study. *BMC Infectious Diseases*.

[9] Watt J. P., O’Brien K. L., Benin A. L. (2004). Invasive pneumococcal disease among Navajo adults, 1989–1998. *Clinical Infectious Diseases*.

[10] Korea Statistical Yearbook (2013). *Annual report on the cause of death statistics 2012*.

[11] Klugman K. P., Madhi S. A., Albrich W. C. (2008). Novel approaches to the identification ofStreptococcus pneumoniaeas the cause of community-acquired pneumonia. *Clinical Infectious Diseases*.

[12] Klugman K. P. (1990). Pneumococcal resistance to antibiotics. *Clinical Microbiology Reviews*.

[13] Song E. K., Lee J. H., Kim N. H. (2005). Epidemiology and clinical features of invasive pneumococcal infections in children. *Korean Journal of Pediatric Infectious Diseases*.

[14] Doern G. V., Richter S. S., Miller A. (2005). Antimicrobial resistance among *Streptococcus pneumoniae* in the United States: have we begun to turn the corner on resistance to certain antimicrobial classes?. *Clinical Infectious Diseases*.

[15] Song J. H., Lee N. Y., Ichiyama S. (1999). Spread of drug-resistant *Streptococcus pneumoniae* in Asian countries: Asian Network for Surveillance of Resistant Pathogens (ANSORP) Study. *Clinical Infectious Diseases*.

[16] Weinstein M. P., Klugman K. P., Jones R. N. (2009). Rationale for revised penicillin susceptibility breakpoints versus *Streptococcus pneumoniae*: coping with antimicrobial susceptibility in an era of resistance. *Clinical Infectious Diseases*.

[17] CLSI (2018). Methods for dilution antimicrobial susceptibility tests for bacteria that grow aerobically. *CLSI Document M07Ed11*.

[18] Cho E. Y., Lee H., Choi E. H. (2014). Serotype distribution and antibiotic resistance of _Streptococcus pneumoniae_ isolated from invasive infections after optional use of the 7-valent conjugate vaccine in Korea, 2006 -2010. *Diagnostic Microbiology and Infectious Disease*.

[19] Vuori-Holopainen E., Peltola H., Kallio M. J. T., for the SE-TU Study Group (2000). Narrow-versus broad-spectrum parenteral antimicrobials against common infections of childhood: a prospective and randomised comparison between penicillin and cefuroxime. *European Journal of Pediatrics*.

[20] Paik J. Y., Choi J. H., Cho E. Y. (2011). Antibiotics Susceptability ofStreptococcus pneumoniaeIsolated from pharynx in healthy Korean children and choice of proper empirical oral antibiotics using pharmacokinetics/pharmacodynamics model. *Korean Journal of Pediatric Infectious Diseases*.

[21] Bae S. M., Lee S. K. (2014). Current state of the serotype distribution and antibiotics resistance of pneumococcal species isolated from the patients in the local community. *KCDC*.

[22] Lee H., Choi E. H., Lee H. J. (2014). Efficacy and effectiveness of extended-valency pneumococcal conjugate vaccines. *Korean Journal of Pediatrics*.

[23] Cho E. Y., Choi E. H., Lee H., Kang J. H., Kim K. H., Lee H. J. Multicentric approach for analysis of serotypes of pneumococcus isolated from invasive infections in Korean children.

[24] Song J. Y., Nahm M. H., Moseley M. A. (2013). Clinical implications of pneumococcal serotypes: invasive disease potential, clinical presentations, and antibiotic resistance. *Journal of Korean Medical Science*.

